# Does Signing Auditor's Reputational Promotion Ease the Financing Constraints of Audited Firms?

**DOI:** 10.1155/2022/3286181

**Published:** 2022-08-03

**Authors:** Chunxia Gu, Rongxia Zhao

**Affiliations:** Shanghai Maritime University, Shanghai, China

## Abstract

Based on the senior certified public accountants selected by the Chinese Institute of Certified Public Accountants and data drawn from China's A-share listed companies from 2014 to 2019, this study studies the influence mechanism of signing auditors' personal reputational promotion on corporate financing constraints. The results show that the improved reputation of signing auditors will help ease the financing constraints faced by companies. Moreover, compared with that of signing auditors from Big Four accounting firms, the improved reputation of signing auditors from non-Big Four firms has a more significant effect on alleviating the financing constraints of enterprises. In addition, private enterprises and small and medium-sized enterprises face more severe financing constraints than state-owned enterprises and large enterprises, and the reputational promotion of signing auditors can better alleviate the financing constraints of the former two types of enterprises. The research conclusions provide theoretical and data-driven support for constructing audit reputation mechanisms in China and improving the financing capabilities of enterprises.

## 1. Introduction

The substitution of formal institutions for informal institutions is a gradual process [1]. While strengthening the legal construction of the market economy, China also actively promotes the construction of reputation mechanisms. The state encourages accounting firms to become increasingly stronger through policies that aim to enhance their reputation [2] and promote the construction of the auditor's reputation mechanism through the selection of senior certified public accountants (CPAs).

Most of the existing studies on audit supervision reputation are conducted from the perspective of accounting firms and analyze the influence mechanism of accounting firms' reputation [3] and its impact on the price of corporate securities [4], audit pricing [5], customer portfolio [6], etc. Previous research on the personal reputation of auditors has been carried out based on the accounting firm's reputation [7, 8] or from the perspective of audit failure. It has been believed that an auditor's tarnished reputation would negatively impact firms, markets, and enterprise financing [6–9]. However, the contagion effect of an auditor's damaged reputation is limited [10], and firm reputation can effectively mitigate the negative impact of individual reputation [9]. Thus, as long as auditors are still qualified, their quasi-rent damage is limited [2]. The limitations of those studies that are based on firm reputation lie in that they neither distinguish individual reputation from organizational reputation, thus showing obvious endogeneity [11], nor discuss the influences of different auditors' reputations in the same firm. Those studies that focused on audit failure were conducted from the perspective of postsupervision and punishment and, therefore, failed to explain the role of the auditor's personal reputation.

The signing auditor is responsible for supervising both the audit work and the production and disclosure of auditing reports. Taking the personal reputation of the signing auditor as the research object can avoid the endogenous problem of the firm's reputation and better demonstrate the role of the reputation mechanism of auditing supervision. The Chinese Institute of Certified Public Accountants (CICPA) has thus far released three senior CPA lists, i.e., in 2010, 2015, and 2017. The resulting changes in auditors' personal reputations provide a good background for studying the impact of personal reputation.

Financing constraints have always been the focus of academic and even practical circles. A large number of studies have shown that financing constraints are one of the major issues restricting the development of Chinese enterprises [12]. So what is the impact of auditor's reputational promotion on the financing constraints of the audited firm? Therefore, this study attempts to explore this issue based on the lists of senior CPAs released by the CICPA in 2010, 2015, and 2017. The results show that the financing constraints of enterprises are significantly reduced when they employ senior CPAs. In addition, senior CPAs who are not from Big Four accounting firms can better alleviate the financing constraints of enterprises. Furthermore, the employment of senior CPAs plays a stronger role in alleviating the financing constraints of private enterprises and small and medium-sized enterprises than those of state-owned and large enterprises. This study helps to clarify the mechanism of auditor reputation and enrich the research on auditor reputation and financing constraints.

## 2. Theoretical Analysis and Research Hypothesis

### 2.1. Signing Auditor Reputational Promotion and Corporate Financing Constraints

The role of supervisors' reputation mechanism depends on enterprises' demand for audits, which can be summarized into three categories, namely, demand for agency cost reduction based on agency theory [13], demand for high-quality information systems and information transmission based on information theory [14, 15], and demand for risk transfer based on insurance theory [16].

The influence of the supervisor's reputation mechanism can be detailed from the following aspects. According to agency theory, auditing reports issued by auditors with a high-level professional reputation can provide high-quality guarantees for corporate financial reports, reduce the information asymmetry between investors and enterprise managers, lower agency costs, and thus alleviate the financing constraints of enterprises [13]. According to information theory, reputable auditors can improve the financial information system of enterprises through their strong professional abilities [15–17]. At the same time, enterprises' employment of auditors with good reputations sends positive signals to the outside world and gains the trust of external investors, which is conducive to alleviating financing constraints and reducing financing costs [18]. According to the insurance hypothesis, in addition to having supervisory function and information value, audits also enable investors to claim civil compensation from auditors in the case of audit failure [16–19]. Thus, investors can transfer financial statement risks through audits, thereby protecting the interests of investors [20] and alleviating the financing constraints of enterprises.

When a senior CPA is hired as a signing auditor, the role of the auditor reputation in helping enterprises alleviate financing constraints becomes obvious. First, the reputation of the senior CPA is proof of the auditor's expertise. The CICPA selects senior CPAs from the best of the best based on their working seniority, professional ability, professional ethics, theoretical research, management experience, etc. Therefore, a senior CPA who is employed by an enterprise can further enhance the supervisory role and information value of the auditing work. Second, the reputational resources of senior CPAs are scarce; once their reputation is damaged, the cost is huge. In 2010, 2015, and 2017, the CICPA announced 395, 609, and 1129 senior CPAs, respectively, which together account for less than 2% of the total number of CPAs in China, and there is no fixed time interval for senior CPA selection. If a senior CPA is paid by a manager to issue a false auditing report, once this has been found out, they will not only lose the title of senior CPA but also be banned from participating in senior CPA selection for life; thus, their reputation will be severely damaged. The scarcity of this reputational resource highlights the professional competence of senior CPAs and enhances the supervisory role and information value. More importantly, such a reputation increases the cost of auditors' audit failures and serves as intangible insurance for investors.

Based on the above analysis, this study believes that the improved reputation of the signing auditor will help alleviate the agency problem of enterprises, increase the information value, strengthen the insurance mechanism, and thus alleviate the financing contract of enterprises. Therefore, this study proposes Hypothesis *H*1 as follows:

 
*H*1: the improved reputation of signing auditors can alleviate the financing constraints faced by listed companies.

The focus of this study is the impact of the personal reputation of the signing auditor, but the auditor's firm is the platform on which the reputation plays its role; thus, the reputational influence mechanism of auditors from different firms should be different. However, there has been little comparative analysis of the differences in the impact of auditors' personal reputation and firms' organizational reputations. Some scholars have analyzed the contagion effect of reputational damage from the perspective of auditor audit failure. It has been found that reputational damage is only contagious among auditors on the same team; the contagion effect on other teams in the firm is limited [10]. At the same time, if the quality control mechanism of the firm is perfect, then the reputation of the firm can effectively reduce the signal transmission value and efficiency of personal reputation [9].

Obviously, a good firm reputation can attenuate the impact of personal reputation. The “Big Four” accounting firms have built a solid brand reputation over the years and have consistently been recognized by the public as representatives of high reputation and quality [21]. Therefore, it is speculated that since firm reputation weakens individual reputation, the reputational promotion of non-Big Four signing auditors is more effective than that of Big Four signing auditors in alleviating the financing constraints of audited firms. Based on the above analysis, this study proposes Hypothesis *H*2 as follows:

 
*H*2: compared with the signing of auditors from Big Four firms, the reputational promotion of signing auditors from non-Big Four firms is more helpful in easing financing constraints for listed companies.

### 2.2. Impact of Enterprise Characteristics

As seen from the above analysis, a signing auditor with the honorary title of senior CPA can effectively alleviate the financing constraints faced by enterprises; however, there are differences in the mitigation effect of financing constraints for companies with different characteristics. This study focuses on the nature of ownership and enterprise scale, which have a great influence on enterprise characteristics.

First, from the perspective of the nature of ownership, this study speculates that the reputational promotion of signing auditors has a significant impact on alleviating the financing constraints of private enterprises. State-owned enterprises tend to have easier access to bank credit, while private enterprises face severe challenges in obtaining bank loans. This is because private enterprises have defects in their own asset structure and financing risks and because financial institutions have stricter loan approval procedures, lower profile quotas, and higher financing cost requirements for private enterprises [22]. In terms of bank loans, state-owned enterprises have a unique advantage of political connection. The government's support for state-owned enterprises can be provided by means such as credit loans from state-controlled banks. From this aspect, the “implicit guarantee” effect of government intervention is more effective than the auditor's reputation. This study, therefore, speculates that the reputational promotion of signing auditors is more conducive to the alleviation of financing constraints faced by private enterprises without implicit government guarantees.

Second, from the perspective of enterprise scale, small and medium-sized enterprises (SMEs) face more severe financing difficulties compared with those of large enterprises. The SMEs are small in scale and have a short establishment time, low quality of information transmission, and less collateral than large enterprises when applying for loans; thus, their external financing friction costs are higher, and they are more prone to financing constraints [23]. Therefore, in this sense, improving the reputation of the signing auditor is more helpful to SMEs. Large enterprises can finance through their own advantages, while SMEs cannot reach a scale that can compete with large enterprises in a short period of time. Therefore, one of the fastest ways for SMEs to finance is to take advantage of the signal transmission function of highly reputable signing auditors. It is theoretically expected that the reputational promotion of signing auditors is more helpful for SMEs than large enterprises with regard to easing financing constraints. Based on the above analysis, this study proposes the following hypotheses:

 
*H*3: compared with state-owned enterprises, the reputational promotion of signing auditors is more helpful for private enterprises with regard to easing financing constraints.
 
*H*4: compared with large enterprises, the reputational promotion of signing auditors is more helpful for SMEs with regard to easing financing constraints.

## 3. Study Design

### 3.1. Sample Selection and Data Sources

The CICPA announced the first batch of senior CPAs in 2010 and the second and third batches in 2015 and 2017, respectively. Data drawn from China A-share listed companies from 2014 to 2019 are used as the research sample; the research sample data are processed as follows: (1) listed companies in the financial industry are excluded; (2) ST and *∗*ST listed companies are excluded; and (3) companies that cannot be calculated by the SA index, which is a measure of financing constraints, are excluded. The basic information, financial data, equity structure, and board information of enterprises are all from the CSMAR database, and the list of senior CPA is from the official website of the CICPA. In addition, winsorization at the 1% level is performed on continuous variables according to the method commonly used in studies of financing constraints.

### 3.2. Variable Definition and Empirical Model

#### 3.2.1. Main Research Variables

*(1) Financing Constraint*. Scholars have improved the measurement methods of financing constraints many times, with the aim of making up for the shortcomings of previous studies. The most representative measurement indicators are the KZ index [24], the WW index [25], and the SA index [26]. Since the KZ index and the WW index need to use some endogenous variables, such as corporate financing leverage and cash flow, in the calculation process, these two indicators have certain defects in regard to measuring corporate financing constraints. To reduce the influence of endogenous variables, this study measures financing constraints with reference to the SA index constructed by Hadlock and Pierce [26]. Only the scale and establishment time of the enterprise are involved in the calculation of the SA index; these variables experience little change over time and are highly exogenous.

*(2) Signing Auditor Reputational Promotion*. To accurately quantify the reputational promotion of signing auditors, the data of CPAs are sorted based on the lists of senior CPAs released by the CICPA in 2010, 2015, and 2017 on the official website of the CICPA and the signing auditors of China A-share listed companies. If the signing auditor of one listed A-share company obtained the honor of senior CPA within the audit year, then a corresponding value is assigned. In particular, signing auditors who received the honorary title of senior CPA in 2010 are assigned a value of 3, those who received the honorary title of senior CPA in 2015 are assigned a value of 2, and those who received the honorary title of senior CPA in 2017 are assigned a value of 1; otherwise, a value of 0 is given. To keep the assignment results consistent with the dependent variable and the control variable on the order of magnitude, they are reduced by a factor of 100 without affecting the reliability of the regression result.

*(3) Model Design*. Referring to relevant studies [19, 27, 28], this study controls for factors such as financial leverage, company growth, profitability, company quality, and ownership structure in the regression. The specific control variables are shown in Table 1. Moreover, to test the hypothesis proposed in this study, the following OLS regression model is constructed:

(1) $$\begin{array}{c} \text{SA}=\alpha_{0}+\alpha_{1}\text{Auditor}+\Sigma \beta_{i}{\text{Control}}_{i}+\Sigma \text{Industry}+\Sigma \text{Year}+\mathrm{\varepsilon ,} \end{array}$$

(2) $$\begin{array}{c} \text{SA}=\alpha_{0}+\alpha_{1}\text{Auditor}+\alpha_{2}\text{Auditor}\times \text{SOE}+\alpha_{3}\text{SOE} \end{array}$$

(3) $$\begin{array}{c} \text{SA}=\alpha_{0}+\alpha_{1}\text{Auditor}+\alpha_{2}\text{Auditor}\times \text{SIZE}+\alpha_{3}\text{SIZE}+\Sigma \beta_{i}{\text{Control}}_{i}\\ +\Sigma \text{Industry}+\Sigma \text{Year}+\varepsilon_{t}. \end{array}$$

In the above formulas, Control is the control variable. Formula (1) tests Hypothesis 1 and uses formula (1) for the group test to test Hypothesis 2. Formula (2) tests Hypothesis 3, and formula (3) tests Hypothesis 4.

## 4. Empirical Results and Analysis

### 4.1. Descriptive Statistics

The calculation result of the SA index is negative; thus, the larger the absolute value is, the more severe the financing constraints of enterprises are. As seen from the data in Table 2, the mean and median of the SA index are −3.801 and −3.798, respectively, which are quite close to each other; this indicates that Chinese listed companies are generally faced with financing constraints and severe financing difficulties. The mean of the dummy variable SOE is 0.358, which means that state-owned enterprises account for more than one-third of the research sample. The average of the shareholding ratio of the largest shareholder (TOP1) is 0.345, and the maximum is 0.900, which indicates that the ownership concentration of China A-share listed companies in the research sample is high. The maximum enterprise scale (SIZE) is 28.640, the minimum is 14.940, and the standard deviation is 1.327, which indicates that there is a considerable gap between the scales of China A-share listed companies. In terms of corporate governance, the mean of independent directors (OUTDIR) is 0.377, and the standard deviation is 0.056, which indicates that the implementation effect of the independent director system of A-share listed companies in China is remarkable and that the gap between listed companies is small. The mean of DUAL is 0.287, which indicates that it is common for the chairman of the board to concurrently serve as the general manager of listed companies in China.

### 4.2. Test of the Effect of Signing Auditor Reputational Promotion on Alleviating Corporate Financing Constraints

In this study, a regression analysis of all sample data is performed first. As shown in the regression results in column (1) of Table 3, after controlling for the commonly used variables that reflect financial leverage, profitability, company growth, corporate governance, and shareholding structure, the regression coefficient of signing auditor reputational promotion (AUDITOR) is significantly positive at the 5% level. This means that the improved reputation of signing auditors does help the listed company alleviate their financing constraints, which verifies Hypothesis *H*1. To test Hypothesis *H*2, this study groups accounting firms according to the type of accounting firm (BIG4) and uses model (1) to test the effect of the reputational promotion of signing auditors on firms' financing constraints. The test results are shown in columns (2) and (3) of Table 3. It can be seen from the test results that the signing auditors from Big Four firms who won the honor of a senior CPA do not have an alleviation effect on corporations' financing constraints, whereas the coefficient of non-Big Four signing auditors is significantly positive at the 5% level. This outcome indicates that, compared with signatory auditors from Big Four firms, the improved reputation of non-Big Four auditors is more conducive to alleviating the financing constraints of listed companies, which verifies Hypothesis *H*2.

From the perspective of control variables, the influence of external supervisors (accounting firms) on corporate financing constraints is first observed. In this study, the Big Four accounting firms are selected as representatives of high-reputation accounting firms. The regression coefficient of BIG4 is positive and significant at the 1% level, which means that hiring reputable accounting firms can greatly alleviate the financing constraints of enterprises. From the perspective of a certain feature of an enterprise, the coefficient of the nature of enterprise property rights (SOE) variable is positive and significant at the 1% level, which means that compared with state-owned enterprises, private enterprises face more severe financing constraints. In terms of the impact of the regional marketization level (Market) on the financing constraints of listed companies, the regression coefficient of Market is significantly positive at the 1% level. This indicates that the higher the degree of regional marketization is, the more conducive it is to reducing financing constraints.

### 4.3. Test of the Influence of Enterprise Characteristics

Table 4 investigates the role of firm ownership nature in the relationship between signing auditor reputational promotion and firm financing constraints. The full-sample regression results in column (1) of Table 4 show that the regression coefficient of the auditor's reputation (AUDITOR) is significantly positive at the 10% level. This means that the reputational promotion of the signing auditor can effectively alleviate the financing constraints of enterprises, which agrees with the abovementioned results. The coefficient of Auditor × Soe is significantly negative at the level of 1%, which means that the nature of enterprise ownership (SOE) will weaken the mitigation effect of signing auditor reputational promotion on corporate financing constraints. Furthermore, the regression coefficient of SOE is significantly positive, which indicates that private enterprises face more serious financing constraints than do state-owned enterprises. Therefore, compared with state-owned enterprises, the improved reputation of signing auditors is more conducive to reducing the financing constraints of private enterprises. The empirical results support Hypothesis *H*3; that is, a signing auditor with the honor of being a senior CPA has a stronger effect on alleviating the financing constraints of private enterprises than those of state-owned enterprises.

Column (2) of Table 4 tests the moderating effect of enterprise scale on signing auditor reputational promotion and financing constraints. It can be seen from the full-sample regression results that the regression coefficient of Auditor×Size is negative and significant at the 1% level. That is, the expansion of the enterprise scale will weaken the effect of the auditor's reputational promotion on the financing constraints of the enterprise to a certain extent. In other words, compared with large enterprises, the reputational promotion of signing auditors is more helpful for SMEs in regard to reducing financing constraints. The test results support Hypothesis *H*4. In summary, the improved reputation of signing an auditor has important theoretical and practical significance for alleviating the financing constraints of enterprises, especially the financing constraints of private enterprises and SMEs.

### 4.4. Influence of Marketization Process

The external market environment has an important impact on enterprises. We use the marketization index to measure the comprehensive external environment of enterprises [29]. The marketization index consists of five aspects: the relationship between government and market, the development of non-state-owned economy, the development of product market, the development of factor market, and the development of the intermediary organization.

We sorted the samples according to the market index, divided them into three groups, deleted the data of the middle group, and tested the high and low groups. The regression results are shown in Table 5. The AUDITOR regression coefficient in column (1) was positive and significant at the 10% level, while the regression result of column (2) was insignificant. It can be seen that for enterprises in regions in a high marketization process, reputational promotion is more conducive to easing the financing constraints. When the level of marketization is higher, the reputation mechanism will be more effective. Once the auditor fails to audit, not only the audit firm will face serious reputation and economic losses, but also auditors themselves will face major reputation damage and professional crisis. Therefore, we need to optimize the external environment of the enterprise so that the reputation mechanism can play a better role.

### 4.5. Robustness Test

To ensure the reliability of the conclusions of this study, several robustness tests are carried out.

First, robustness tests on alternative variables of signing auditor reputational promotion are performed. To exclude the influence of subjective assignment on the research conclusion, the values of 0, 1, 2, and 3 initially assigned to auditor reputational promotion (AUDITOR) are replaced by values of 0 and 1. The regression results are shown in Table 6. The regression results also support the hypothesis, which indicates that the conclusions of this study remain robust.

Second, different conclusions may be drawn when different indicators are selected to measure the financing constraints of enterprises. To test whether the research conclusions are sensitive to the measurement method of corporate financing constraints, this study uses the WW index to replace the SA index. The variables used in the calculation of the WW index are relatively comprehensive in economic significance. In the calculation of this index, not only the variables that reflect the financial characteristics of the enterprise but also those that reflect the external industry factors of the enterprise are considered. Generally, the larger the value of this index is, the more serious the financing constraints are. As shown in Table 7 (column 6 shows the result of Hypothesis *H*1 based on KZ index), the WW index and KZ index regression results are basically consistent with the SA index regression results and support the hypothesis, which indicates that the research conclusions of this study are not affected by the choice of the measurement index of financing constraints.

Third, to further ensure the validity of the study results and in view of the possible endogeneity problems, the lagged signatory auditor reputation (L. AUDITOR) is used as an independent variable. The regression results are shown in Table 8. The research results show that the previous conclusions are still valid after controlling for the above problems, which indicates that the major research conclusions of this study have good robustness.

## 5. Conclusions and Implications

The “Enron Incident” that occurred in the United States in 2001 was a devastating blow to Arthur Andersen, which was one of the Big Five accounting firms at that time; the incident also raised serious concerns about the reputation of auditors. In 2002, the “Guangxia (Yinchuan) Incident” in China caused the Zhongtianqin accounting firm to face the same situation as that faced by Arthur Andersen and a shock to China's capital market. Since then, an increasing number of Chinese scholars have begun to study auditor reputation. The Chinese government also actively promotes the construction and development of an auditor's reputation mechanism to combine the “internal force” (auditor reputation system) with the “external force” (legal system). The auditor's reputation system can better regulate the auditor's behavior and improve audit quality. Most of the current studies on auditor reputation are analyzed from the firm reputation. The impact of auditor reputation on enterprises is mainly analyzed from the perspective of auditor punishment. The lists of senior CPAs published by the CICPA since 2010 have provided a good research background on the reputational promotion of auditors.

Therefore, based on the data of China's A-share listed companies from 2014 to 2019 and the three lists of senior CPAs published by CICPA, this study examined the mitigation effect of the reputational promotion of signing auditors on corporate financing constraints. The research results show that the reputational promotion of signing auditors can significantly alleviate the financing constraints of enterprises. The research results provide theoretical and data-driven support for China to promote the construction of an auditor reputation mechanism. Moreover, to investigate the influence at the firm level, this study conducted a group test on the accounting firms where the signing auditors work. All the samples were divided into two sample groups for regression according to whether they are Big Four accounting firms. The regression results show that the reputational promotion of non-Big Four signing auditors can significantly reduce the financing constraints of enterprises, while the reputational promotion of Big Four auditors has no significant effect on alleviating financing constraints. While organizational reputation can weaken the influence of individual reputation, it is particularly necessary for a group with a weak organizational reputation to establish an individual reputation. In addition, this study, through the two most representative corporate characteristics, namely, the nature of property rights and the enterprise scale, further studied the role of corporate characteristics in the relationship between auditor reputational promotion and corporate financing constraints. The results show that the reputational promotion of signing auditors can better ease the financing constraints of private enterprises and small and medium-sized enterprises compared with those of state-owned enterprises and large enterprises.

The research results partly verify the positive role of China's auditor's reputational system and provide new ideas for private enterprises and SMEs to ease their financing constraints. However, we acknowledge some limitations of our study. We studied listed Chinese companies, and the results are likely to be relatively stable only in similar regions and countries. Also, we only studied the influence of auditor's reputational promotion on the financing constraints of the audited enterprises. However, the role of the external supervision reputation mechanism is more extensive and profound. In the future, we may need to consider other aspects of the audited companies (like investment decision and innovation). Also, future research might investigate whether internal governance and external economic and political conditions affect the stability of the results. In addition, we only tested data from Chinese enterprises in this study. In the future, we can explore the issue based on data from different countries or regions for comparative research.

## Figures and Tables

**Table 1:** Description of related variables.

Variable		Symbol	Definition
Dependent variable	SA index	SA	−0.737 × SIZE + 0.043 × SIZE^2^ − 0.04 × AGE
	WW index	WW	−0.091 × CF_1_ − 0.062 × DIVPOS + 0.021 × TLTD − 0.044 × LNTA + 0.102 × ISG − 0.035 × SG
	KZ index	KZ	−1.00191 × CF_2_ + 3.13919 × TLTD − 39.36780 × TDIV − 1.31476 × CASH + 0.28264 × Tobin's Q

Independent variable	Signing auditor reputational promotion	Auditor	A dummy variable that is assigned a value of 3 if the signing auditor won the honorary title of senior CPA in 2010, 2 if the auditor won in 2015, 1 if the auditor won in 2017, and 0 otherwise
Moderator variable	Big Four accounting firms in the world	BIG4	A dummy variable that is assigned a value of 1 when the accounting firm is one of the BIG4 firms and 0 otherwise
	Enterprise scale	SIZE	Natural logarithm of the total assets of an enterprise at the end of the period
	The nature of enterprise property rights	SOE	A dummy variable, which is assigned a value of 1 if the enterprise is state-owned and 0 otherwise

Control variable	Ratio of liabilities to assets	LEV	Total liabilities/total assets
	Cash flow from operations	CFO	Net cash flow from operating activities/total assets
	Corporate growth	Tobin's Q	(Market value of equity + market value of net debt)/total assets at the end of the period
	Return on assets	ROA	Net profit/total average assets
	Company age	AGE	The natural logarithm of the number of years the company has been established
	Shareholding ratio of the largest shareholder	TOP1	Shareholding ratio of the largest shareholder disclosed in the corporate annual report
	Board of directors	BSIZE	The natural logarithm of the number of board members of a company
	Independent directors	OUTDIR	Number of independent directors/total number of directors
	Duality of general manager and chairman	DUAL	A dummy variable, which is assigned a value of 1 when the chairman and the general manager are the same person and 0 otherwise

Data source: collected and sorted by the authors. *Note*. SIZE = natural logarithm for the total assets of an enterprise at the end of the period; AGE = observed year-year of the listed; CF_1_ = operating net cash flow; DIVPOS is a dummy variable, which is 1 if the firm pays dividends and 0 otherwise; TLTD = long-term liabilities/total assets; ISG is the industry sale growth rate; SG = operating revenue growth; CF_2_ = operating net cash flow/total assets; TLTD = total liabilities/total assets; TDIV = cash dividend/total assets; CASH is cash holdings/total assets.

**Table 2:** Descriptive statistics of major variables.

	Mean	Minimum	Median	Maximum	SD
SA index	−3.801	−5.543	−3.798	−1.455	0.253
LEV	0.414	0.00840	0.402	4.026	0.206
ROA	0.054	−1.535	0.053	0.767	0.080
CFO	0.048	−0.888	0.047	0.876	0.074
SOE	0.358	0.000	0.000	1.000	0.479
SIZE	22.230	14.940	22.060	28.640	1.327
TOP1	0.345	0.003	0.326	0.900	0.148
BSIZE	2.119	1.099	2.197	2.996	0.200
OUTDIR	0.377	0.200	0.364	0.800	0.056
DUAL	0.287	0.000	0.000	1.000	0.452

Data source: collected and sorted by the authors.

**Table 3:** Signing auditor reputational promotion and corporate financing constraints.

	(1)	(2)	(3)
	Full sample	BIG4 = 1	BIG4 = 0
AUDITOR	0.269^∗∗^	−0.916	0.262^∗∗^
	(0.040)	(0.504)	(0.018)

LEV	0.043^∗∗∗^	0.523^∗∗∗^	0.023^∗∗∗^
	(0.000)	(0.000)	(0.000)

ROA	−0.029^∗∗^	0.287	−0.019^∗^
	(0.034)	(0.134)	(0.091)

CFO	0.020	0.484^∗∗∗^	0.005
	(0.154)	(0.000)	(0.710)

AGE	−0.663^∗∗∗^	−0.764^∗∗∗^	−0.647^∗∗∗^
	(0.000)	(0.000)	(0.000)

SOE	0.017^∗∗∗^	0.085^∗∗∗^	0.008^∗∗∗^
	(0.000)	(0.000)	(0.000)

Tobin's Q	0.004^∗∗∗^	−0.033^∗∗∗^	0.004^∗∗∗^
	(0.000)	(0.000)	(0.000)

TOP1	0.062^∗∗∗^	0.180^∗∗∗^	0.051^∗∗∗^
	(0.000)	(0.000)	(0.000)

BSIZE	0.074^∗∗∗^	0.318^∗∗∗^	0.047^∗∗∗^
	(0.000)	(0.000)	(0.000)

OUTDIR	0.319^∗∗∗^	0.899^∗∗∗^	0.159^∗∗∗^
	(0.000)	(0.000)	(0.000)

DUAL	0.011^∗∗∗^	−0.006	0.011^∗∗∗^
	(0.000)	(0.769)	(0.000)

BIG4	0.151^∗∗∗^		
	(0.000)		

Market	0.002^∗∗∗^	0.030^∗∗∗^	−0.0004
	(0.000)	(0.000)	(0.367)

Industry	Control	Control	Control
Year	Control	Control	Control
Constant	−2.313^∗∗∗^	−3.424^∗∗∗^	−2.198^∗∗∗^
	(0.000)	(0.000)	(0.000)

*N*	16536	952	15584
*R* [2]	0.770	0.711	0.817

*Note. P* values are in parentheses, and ^∗∗∗^, and ^∗∗∗^ indicate significance at the 10%, 5%, and 1% levels, respectively. Data source: collected and sorted by the authors.

**Table 4:** Tests of the influence of enterprise characteristics.

	(1)	(2)
	Full sample	Full sample
AUDITOR	0.354^∗∗^	7.417^∗∗∗^
	(0.045)	(0.000)

SOE	0.026^∗∗∗^	
	(0.000)	

Auditor × Soe	−0.514^∗^	
	(0.061)	

SIZE		0.008^∗∗∗^
		(0.000)

Auditor × Size		−0.329^∗∗∗^
		(0.000)

LEV	0.059^∗∗∗^	−0.022^∗∗∗^
	(0.000)	(0.000)

ROA	−0.012	−0.034^∗∗∗^
	(0.412)	(0.000)

AGE	−0.664^∗∗∗^	−0.483^∗∗∗^
	(0.000)	(0.000)

CFO	0.050^∗∗∗^	0.023^∗∗∗^
	(0.330)	(0.000)

Tobin's Q	0.004^∗∗∗^	0.004^∗∗∗^
	(0.000)	(0.000)

TOP1	0.084^∗∗∗^	0.039^∗∗∗^
	(0.000)	(0.000)

BSIZE	0.090^∗∗∗^	0.003
	(0.000)	(0.579)

OUTDIR	0.371^∗∗∗^	0.016
	(0.000)	(0.245)

DUAL	0.009^∗∗∗^	0.005^∗∗∗^
	(0.000)	(0.000)

Market	0.004^∗∗∗^	0.003^∗∗∗^
	(0.000)	(0.001)

Industry	Control	Control
Year	Control	Control
Constant	−2.390^∗∗∗^	−2.648^∗∗∗^
	(0.000)	(0.000)

*N*	16536	16536
*R* [2]	0.752	0.737

*Note. P* values are in parentheses, and ^∗∗∗^, and ^∗∗∗^ indicate significance at the 10%, 5%, and 1% levels, respectively. Data source: collected and sorted by the authors.

**Table 5:** Test of the influence of marketization process.

	(1)	(2)
AUDITOR	0.003^∗^	0.004
	(0.097)	(0.184)

SOE	0.003	0.039^∗∗∗^
	(0.304)	(0.000)

LEV	0.058^∗∗∗^	0.087^∗∗∗^
	(0.000)	(0.000)

ROA	0.031	0.017
	(0.113)	(0.452)

AGE	−0.632^∗∗∗^	−0.695^∗∗∗^
	(0.000)	(0.000)

CFO	0.0134	−0.010
	(0.507)	(0.714)

Tobin's Q	0.004^∗∗∗^	0.004^∗∗∗^
	(0.000)	(0.008)

TOP1	0.061^∗∗∗^	0.075^∗∗∗^
	(0.000)	(0.000)

BSIZE	0.041^∗∗∗^	0.108^∗∗∗^
	(0.000)	(0.000)

OUTDIR	0.157^∗∗∗^	0.429^∗∗∗^
	(0.000)	(0.000)

DUAL	0.006	0.014^∗∗∗^
	(0.106)	(0.000)

Industry	Control	Control
Year	Control	Control
Constant	−2.219^∗∗∗^	−2.306^∗∗∗^
	(0.000)	(0.000)

*N*	5539	5366
	0.796	0.742

*Note. P* values are in parentheses, and ^∗∗∗^ and ^∗∗∗^ indicate significance at the 10%, 5%, and 1% levels, respectively. Data source: collected and sorted by the authors.

**Table 6:** Robustness tests on alternative variable of signing auditor reputational promotion.

	(1)	(2)	(3)	(4)	(5)
		BIG4 = = 0	BIG4 = = 1		
AUDITOR	0.549^∗∗^	0.463^∗∗^	−0.874	0.320^∗∗^	8.576^∗∗∗^
	(0.026)	(0.028)	(0.675)	(0.026)	0

Auditor × Soe (SIZE)				−0.362^∗^	−0.374^∗∗∗^
				(0.098)	(0.000)

SIZE					0.008^∗∗∗^
					(0.000)

SOE	0.017^∗∗∗^	0.00767^∗∗∗^	0.085^∗∗∗^	−0.023^∗∗∗^	
	(0.000)	(0.000)	(0.000)	(0.000)	

LEV	0.043^∗∗∗^	0.022^∗∗∗^	0.523^∗∗∗^	0.041^∗∗∗^	−0.022^∗∗∗^
	(0.000)	(0.000)	(0.000)	(0.000)	(0.000)

ROA	−0.029^∗∗^	−0.020^∗^	0.293	0.026^∗∗∗^	−0.034^∗∗∗^
	(0.033)	(0.090)	(0.127)	(0.000)	(0.000)

AGE	−0.663^∗∗∗^	−0.646^∗∗∗^	−0.764^∗∗∗^	0.077^∗∗∗^	−0.484^∗∗∗^
	(0.000)	(0.000)	(0.000)	(0.000)	(0.000)

CFO	0.021	0.005	0.481^∗∗∗^	0.019^∗∗∗^	0.023^∗∗∗^
	(0.152)	(0.707)	(0.000)	(0.000)	(0.000)

Tobin's Q	0.004^∗∗∗^	0.004^∗∗∗^	−0.034^∗∗∗^	0.004^∗∗∗^	0.004^∗∗∗^
	(0.000)	(0.000)	(0.000)	(0.000)	(0.000)

TOP1	0.062^∗∗∗^	0.051^∗∗∗^	0.180^∗∗∗^	0.045^∗∗∗^	0.039^∗∗∗^
	(0.000)	(0.000)	(0.000)	(0.000)	(0.000)

BSIZE	0.074^∗∗∗^	0.047^∗∗∗^	0.319^∗∗∗^	0.003	0.003
	(0.000)	(0.000)	(0.000)	(0.578)	(0.570)

OUTDIR	0.319^∗∗∗^	0.159^∗∗∗^	0.898^∗∗∗^	0.004	0.016
	(0.000)	(0.000)	(0.000)	(0.767)	(0.231)

DUAL	0.011^∗∗∗^	0.011^∗∗∗^	−0.006	0.004^∗∗∗^	0.005^∗∗∗^
	(0.000)	(0.000)	(0.793)	(0.001)	(0.000)

Market	0.002^∗∗∗^	−0.0004	0.031^∗∗∗^	0.001	0.003^∗∗∗^
	(0.000)	(0.377)	(0.000)	(0.650)	(0.000)

BIG4	0.151^∗∗∗^				
	(0.000)				

Year	Control	Control	Control	Control	Control
Industry	Control	Control	Control	Control	Control
Constant	−2.313^∗∗∗^	−2.198^∗∗∗^	−3.427^∗∗∗^	−3.549^∗∗∗^	−2.641^∗∗∗^
	(0.000)	(0.000)	(0.000)	(0.000)	(0.000)

*N*	16536	15584	952	16536	16536
*R* ^2^	0.77	0.817	0.71	0.81	0.769

*Note. P* values are in parentheses, and ^∗^, ^∗∗^, and ^∗∗∗^ indicate significance at the 10%, 5%, and 1% levels, respectively. Data source: collected and sorted by the authors.

**Table 7:** Robustness test on alternative variables of financing constraints.

	(1)	(2)	(3)	(4)	(5)	(6)
		BIG4 = = 0	BIG4 = = 1			
AUDITOR	−0.107^∗^	−0.116^∗^	0.208	−0.178^∗^	−0.069^∗^	−0.019^∗∗^
	(0.099)	(0.076)	(0.528)	(0.050)	(0.099)	(0.045)

Auditor × Soe(SIZE)				0.277^∗∗^	0.0001^∗∗∗^	
				(0.038)	(0.000)	

SIZE					−0.047^∗∗∗^	
					(0.000)	

SOE	−0.011^∗∗∗^	0.010^∗∗∗^	0.021^∗∗∗^	−0.015^∗∗∗^		0.190^∗∗∗^
	(0.000)	(0.000)	(0.000)	(0.000)		(0.000)

LEV	−0.110^∗∗∗^	0.105^∗∗∗^	0.169^∗∗∗^	−0.117^∗∗∗^	0.0139^∗∗∗^	3.989^∗∗∗^
	(0.000)	(0.000)	(0.000)	(0.000)	(0.000)	(0.000)

ROA	−0.266^∗∗∗^	0.269^∗∗∗^	0.368^∗∗∗^	−0.274^∗∗∗^	−0.165^∗∗∗^	−3.765^∗∗∗^
	(0.000)	(0.000)	(0.000)	(0.000)	(0.000)	(0.000)

AGE	0.008^∗∗∗^	0.005^∗∗∗^	0.035^∗∗∗^	0.008^∗∗∗^	0.005^∗∗∗^	0.050^∗∗^
	(0.000)	(0.000)	(0.000)	(0.000)	(0.000)	(0.031)

CFO	−0.081^∗∗∗^	0.076^∗∗∗^	0.147^∗∗∗^	−0.094^∗∗∗^	−0.069^∗∗∗^	−3.650^∗∗∗^
	(0.000)	(0.000)	(0.000)	(0.000)	(0.000)	(0.000)

Tobin's Q	0.008^∗∗∗^	0.007^∗∗∗^	0.033^∗∗∗^	0.008^∗∗∗^	0.001^∗∗∗^	0.099^∗∗∗^
	(0.000)	(0.000)	(0.000)	(0.000)	(0.000)	(0.000)

TOP1	−0.032^∗∗∗^	0.031^∗∗∗^	0.033^∗∗∗^	−0.041^∗∗∗^	−0.009^∗∗∗^	−0.731^∗∗∗^
	(0.000)	(0.000)	(0.000)	(0.000)	(0.000)	(0.000)

BSIZE	−0.058^∗∗∗^	0.057^∗∗∗^	0.054^∗∗∗^	−0.064^∗∗∗^	0.0005	−0.110^∗∗^
	(0.000)	(0.000)	(0.000)	(0.000)	(0.810)	(0.014)

OUTDIR	−0.121^∗∗∗^	0.107^∗∗∗^	0.140^∗∗∗^	−0.146^∗∗∗^	0.020^∗∗∗^	0.238
	(0.000)	(0.000)	(0.000)	(0.000)	(0.000)	(0.114)

DUAL	0.004^∗∗∗^	0.004^∗∗∗^	0.006	0.004^∗∗∗^	−0.001	−0.071^∗∗∗^
	(0.000)	(0.000)	(0.268)	(0.000)	(0.121)	(0.000)

Market	−0.002^∗∗∗^	0.001^∗∗∗^	0.005^∗∗∗^	−0.003^∗∗∗^	−0.001^∗∗∗^	−0.005
	(0.000)	(0.000)	(0.000)	(0.000)	(0.000)	(0.157)

BIG4	−0.056^∗∗∗^					−0.081^∗∗∗^
	(0.000)					(0.000)

Year	Control	Control	Control	Control	Control	Control
Industry	Control	Control	Control	Control	Control	Control
Constant	−0.782^∗∗∗^	0.787^∗∗∗^	0.815^∗∗∗^	−0.747^∗∗∗^	0.0171^∗^	1.737^∗∗∗^
	(0.000)	(0.000)	(0.000)	(0.000)	(0.093)	(0.000)

*N*	10933	10192	741	10933	10933	15145
*R* ^2^	0.458	0.389	0.542	0.419	0.455	0.611

*Note. P* values are in parentheses, and ^∗^, ^∗∗^, and ^∗∗∗^ indicate significance at the 10%, 5%, and 1% levels, respectively. Data source: collected and sorted by the authors.

**Table 8:** Robustness test based on lagged signatory auditor reputation.

	(1)	(2)	(3)
		BIG4 = = 0	BIG4 = = 1
AUDITOR	0.284^∗^	0.259^∗∗^	−1.372
	(0.055)	(0.029)	(0.352)

SOE	0.016^∗∗∗^	0.013^∗∗∗^	0.082^∗∗∗^
	(0.000)	(0.000)	(0.000)

LEV	0.049^∗∗∗^	0.052^∗∗∗^	0.573^∗∗∗^
	(0.000)	(0.000)	(0.000)

ROA	0.004	−0.017	0.512^∗∗^
	(0.795)	(0.168)	(0.022)

AGE	−0.696^∗∗∗^	0.678^∗∗∗^	0.819^∗∗∗^
	(0.000)	(0.000)	(0.000)

CFO	−0.002	0.008	0.461^∗∗∗^
	(0.882)	−0.571	(0.000)

Tobin's Q	0.011^∗∗∗^	0.011^∗∗∗^	0.035^∗∗∗^
	(0.000)	(0.000)	(0.000)

TOP1	0.061^∗∗∗^	0.056^∗∗∗^	0.179^∗∗∗^
	(0.000)	(0.000)	(0.000)

BSIZE	0.080^∗∗∗^	0.064^∗∗∗^	0.310^∗∗∗^
	(0.000)	(0.000)	(0.000)

OUTDIR	0.322^∗∗∗^	0.177^∗∗∗^	0.948^∗∗∗^
	(0.000)	(0.000)	(0.000)

DUAL	0.010^∗∗∗^	0.009^∗∗∗^	−0.018
	(0.000)	(0.000)	(0.481)

Market	0.002^∗∗∗^	−0.0001	0.032^∗∗∗^
	(0.000)	(0.871)	(5.43)

BIG4	0.149^∗∗∗^		
	(0.000)		

Year	Control	Control	Control
Industry	Control	Control	Control
Constant	−2.200^∗∗∗^	2.198^∗∗∗^	3.323^∗∗∗^
	(0.000)	(0.000)	(0.000)

*N*	13108	12334	774
*R* ^2^	0.774	0.816	0.701

*Note. P* values are in parentheses, and ^∗^, ^∗∗^, and ^∗∗∗^ indicate significance at the 10%, 5%, and 1% levels, respectively. Data source: collected and sorted by the authors.

## Data Availability

Data are included within the article.
